The article "EEG-Based Spectral Dynamic in Characterization of Poststroke Patients with Cognitive Impairment for Early Detection of Vascular Dementia" was published in 2022. Journal: J Healthc Eng.

# EEG-Based Spectral Dynamic in Characterization of Poststroke Patients with Cognitive Impairment for Early Detection of Vascular Dementia

**DOI:** 10.1155/2022/5666229

**Published:** 2022-11-19

**Authors:** Sugondo Hadiyoso, Paulus Anam Ong, Hasballah Zakaria, Tati Latifah E. Rajab

**Affiliations:** ^1^School of Electrical Engineering and Informatics, Bandung Institute of Technology, Bandung, Indonesia; ^2^School of Applied Science, Telkom University, Bandung, Indonesia; ^3^Departement of Neurology, Faculty of Medicine, Padjadjaran University, Dr. Hasan Sadikin General Hospital, Bandung, Indonesia

## Abstract

One common type of vascular dementia (VaD) is poststroke dementia (PSD). Vascular dementia can occur in one-third of stroke patients. The worsening of cognitive function can occur quickly if not detected and treated early. One of the potential medical modalities for observing this disorder by considering costs and safety factors is electroencephalogram (EEG). It is thought that there are differences in the spectral dynamics of the EEG signal between the normal group and stroke patients with cognitive impairment so that it can be used in detection. Therefore, this study proposes an EEG signal characterization method using EEG spectral power complexity measurements to obtain features of poststroke patients with cognitive impairment and normal subjects. Working memory EEGs were collected and analyzed from forty-two participants, consisting of sixteen normal subjects, fifteen poststroke patients with mild cognitive impairment, and eleven poststroke patients with dementia. From the analysis results, it was found that there were differences in the dynamics of the power spectral in each group, where the spectral power of the cognitively impaired group was more regular than the normal group. Notably, (1) significant differences in spectral entropy (SpecEn) with a *p* value <0.05 were found for all electrodes, (2) there was a relationship between SpecEn values and the severity of dementia (SpecEn_Dem_ < SpecEn_MCI_ < SpecEn_Normal_), and (3) a post hoc multiple comparison test showed significant differences between groups at the F7 electrode. This study shows that spectral complexity analysis can discriminate between normal and poststroke patients with cognitive impairment. For further studies, it is necessary to simulate performance validation so that the proposed approach can be used in the early detection of poststroke dementia and monitoring the development of dementia.

## 1. Introduction

Vascular dementia (VaD) is one of the most common types of dementia after Alzheimer's dementia (AD) [1]. Vascular dementia accounts for about 20% of dementia cases worldwide [2]. VaD is a form of cognitive impairment associated with cerebrovascular disease [3]. Stroke is the vascular disease that is the second most commonly associated with VaD. Impaired cognitive function due to stroke is often underestimated compared to motoric dysfunction [4]. It is thought that cognitive impairment will also contribute to the quality of the patient's health problems and lead to dependence on the people around them.

The article "EEG-Based Spectral Dynamic in Characterization of Poststroke Patients with Cognitive Impairment for Early Detection of Vascular Dementia" was published in 2022. Journal: J Healthc Eng.

Based on previous studies, stroke patients will develop 15–30% of dementia three months after stroke, and about 20–25% will develop delayed dementia [5]. Risk factors can potentially increase with age [6]. Decreased cognitive function due to dementia can have a broad impact, including decreased social activities in daily life and increased costs for families, communities, and the government [7] so early detection is needed to prevent the worsening of dementia, which may occur quickly.

The diagnostic process of VaD is complex because it must go through the stages of clinical diagnosis of cognitive impairment that is severe enough to meet the criteria for dementia, and it must be proven that the dementia is the result of cerebrovascular events, including stroke, as evidenced by brain imaging [8]. One alternative cognitive screening test that can be used considering cost and time is the Mini-Mental State Examination (MMSE) or the Montreal Cognitive Assessment (MoCA) [9]. Furthermore, the diagnosis of dementia can be supported by examining genetic polymorphisms, cerebrospinal fluid, and microRNA profiling [10–12]. Medical imaging techniques are also essential instruments for establishing poststroke dementia. Medical imaging modalities have high sensitivity and specificity for detecting pathological changes, including small blood vessel damage that causes cognitive impairment [13]. However, genetic and medical imaging methods require specific equipment that is relatively expensive, complex in installation, not always available, and may pose risks if performed regularly in a short time. One of the biomarkers that can be an alternative in studying brain function related to dementia is the electroencephalogram (EEG), which is supported by quantitative measurements [14].

Over the past several decades, quantitative EEG (QEEG) has been used to complete the criteria for dementia. Recently, QEEG research on dementia has focused on early detection, evaluation of severity, and discrimination of dementia type [15, 16]. Most studies characterize or detect Alzheimer's dementia (AD) based on the EEG. Meanwhile, poststroke dementia has not been widely explored. Considering the risk of stroke, which continues to increase every year, is followed by the risk of dementia, it is necessary to study the detection of poststroke dementia using EEG. Recently, a previous study was conducted to characterize EEG signals from normal subjects and poststroke patients with cognitive impairment. This study showed different power spectral characteristics between normal and poststroke with cognitive impairment [17]. Other studies on the detection of poststroke dementia based on EEG are also reported in [18, 19]. In their study, measurement of signal complexity was used to extract EEG features from normal subjects, stroke-related mild cognitive impairment (MCI), and VaD.

The article "EEG-Based Spectral Dynamic in Characterization of Poststroke Patients with Cognitive Impairment for Early Detection of Vascular Dementia" was published in 2022. Journal: J Healthc Eng.

One of the degrees of complexity proposed in the study [19] is spectral entropy (SpecEn), which represents a measure of EEG spectral dynamics. The degree of EEG spectral dynamics is thought to have a close relationship with a cognitive function where there is a signal pattern transition when responding to a stimulus. The study [19] reported that SpecEn in the group with cognitive impairment was lower than in the normal group. However, in this study, no significant difference was found (*p* < 0.05) in all EEG channels with a frequency range (1–60 Hz). It is thought that in the EEG spectral analysis, high-frequency-band activities play a more important role in emotion than cognitive function, as reported in [20].

Therefore, this study proposes a characterization of EEG signals in poststroke patients with cognitive impairment using the SpecEn approach at a different frequency range from previous studies. In this study, SpecEn was measured in the frequency range of 1–30 Hz as a representation of delta, theta, alpha, and beta waves. The EEG wave pattern in this band is more representative of resting, awake, focused, and thinking conditions. Thus, it is hoped that significant differences will be found between the observed groups. This study involved forty-two participants consisting of sixteen normal subjects, fifteen poststroke patients with mild cognitive impairment, and eleven poststroke patients with dementia. SpecEn measurements were performed during working memory EEG recordings. This study obtained the spectral dynamics characteristics of the EEG signal and the significant differences between groups. The proposed method is expected to be used for feature extraction combined with machine learning for the early detection of poststroke dementia.

The paper is structured as follows: Section 2 contains descriptions of materials and methods, including EEG recording, signal preprocessing, spectral entropy, and statistical methods.  Section 3 contains simulation results, including signal preprocessing results, SpecEn measurement results for each group, and the calculation of significant differences, followed by a discussion.  Section 4 contains the conclusions of the study, limitations, and future work.

The article "EEG-Based Spectral Dynamic in Characterization of Poststroke Patients with Cognitive Impairment for Early Detection of Vascular Dementia" was published in 2022. Journal: J Healthc Eng.

## 2. Materials and Methods

The stages of EEG spectral dynamics measurement and analysis in this study are shown in Figure 1. It includes EEG recording, signal preprocessing, SpecEn calculation, and a significance test on each EEG channel. Details of the stages and methods used in this study are presented in the following subsections.

### 2.1. Subject Criteria and EEG Recording

The type of research used is a quantitative study with a case-control study design with a total of 42 participants consisting of 16 subjects with normal categories, 15 subjects with ischemic stroke patients without dementia (MCI), and 11 subjects with ischemic stroke patients with dementia. Recruitment of participants in this study was conducted at Hasan Sadikin General Hospital, Bandung, Indonesia, after obtaining ethical approval no. LB.02.01/X.6.5/272/2019. All participants are willing to be included in this study by filling out the informed consent. The subject criteria used in this study were based on recommendations. They were selected by a neurologist (Neurobehavioral Consultant), the Indonesian Neurologist Association (PERDOSSI), after a clinical examination, neuropsychology, and brain imaging (CT-scan) were carried out.

Normal subjects were recruited with the following criteria: healthy, no indication of neurological and physiological disorders, and never had a severe brain injury. Meanwhile, the recruited poststroke patients had the following criteria: a stroke at least in the last three months and a complaint of cognitive impairment. Exclusion criteria for both sample groups: subjects with aphasia; From anamnesis, there were no sensory disturbances in hearing, vision, movement disorders, and a history of cerebral diseases such as epilepsy, severe head injury, multiple sclerosis, brain tumors, history of brain surgery, alcoholism by a neurologist.

Cognitive function status was confirmed using the MoCA Indonesian Version (MoCA-INA) test and interviews by psychologists and neurologists. The MoCA score is greater than 26 normal considerations. MoCA less than 19 and having disturbances in basic and instrumental daily activities are poststroke patients with dementia. Meanwhile, for patients with mild vascular cognitive impairment, the MoCA-INA score is between 19 and 25, and there are no disturbances in basic daily activities or mild disturbances in daily instrumental activities. The demographic data in this study are presented in Table 1.

EEG recording was carried out at the diagnostic center of Hasan Sadikin General Hospital using a 19-channel Cadwell Easy III amplification system. The tapped EEG channels refer to 10–20 systems, including Fp1, Fp2, F7, F3, Fz, F4, F8, T3, C3, Cz, C4, T4, T5, P3, Pz, P4, T6, O1, and O2 with reference channels A1 and A2. Cadwell EEG has a sampling frequency of 250 Hz, a sensitivity of 0.5 mV, 18 bit ADC resolution, and the ability to reject noise >110 dB at a frequency of 50–60 Hz. The recording is done in a comfortable, closed room with low light intensity and a minimum sound level. During the recording, the subject lies down on a bed. All participants were given a stimulus by the operator to memorize five familiar words (“face,” “silk,” “mosque,” “orchid,” and “red”) and then mentioned these words. EEG recordings at rest with closed eyes at the time before and after the stimulus were then ignored. This study has received ethical approval from the hospital ethics committee, and all participants agreed to be included in this study by filling out an informed consent form.

The article "EEG-Based Spectral Dynamic in Characterization of Poststroke Patients with Cognitive Impairment for Early Detection of Vascular Dementia" was published in 2022. Journal: J Healthc Eng.

### 2.2. EEG Signal Processing Stages

The aim of the EEG signal processing in this study is to obtain the spectral complexity features of each observed group. The signal processing stages are presented in Figure 1. The first step is preprocessing, including noise removal for 19 channels of EEG signal in the time domain. The main objective is to eliminate low- and high-frequency noise, which are common and dominant due to eyeball movement, blinking, jaw muscle activity, and line noise [21]. The ICA-based decomposition method is applied to observe the noise component. The EEG electrode, suspected of containing a large amount of noise, becomes the basis for elimination. The decomposition process, electrode selection containing noise, and elimination were carried out using the EEGLAB toolbox. At this stage, filtering is also carried out using a digital band-pass filter at a frequency of 1 to 30 Hz. The next step is the quantization of signal complexity parameters using SpecEn. SpecEn value difference test is then applied to observe the significance value. Details of the proposed method are described in the following subsections.

### 2.3. Preprocessing Stage

Artifact noise is generally caused by the influence of limb movements, especially eyeball movement and eye blinking. Another form of noise is baseline wandering, which is often present at low frequencies and causes changes in the baseline signal. Line noise occurs because the operating frequency of the power source is in the 50–60 Hz range. Meanwhile, muscle noise will interfere at high frequencies due to electromyography (EMG) signals around the jaws of the mouth, which have frequency characteristics between 30 and 400 Hz. Therefore, two approaches are used at this stage to remove the noise, including Independent Component Analysis (ICA) and a digital filter with a cut-off frequency of 1–30 Hz. The ICA process is carried out using the EEGLAB toolbox in MATLAB [22].

The article "EEG-Based Spectral Dynamic in Characterization of Poststroke Patients with Cognitive Impairment for Early Detection of Vascular Dementia" was published in 2022. Journal: J Healthc Eng.

The denoising process using ICA is principally a decomposition that involves changing the linear basis of the data collected at each electrode and then transforming it spatially. Each row of the data activation matrix provides the time direction of the activity of one component process that is spatially filtered from the EEG electrode data. In the case of ICA parsing, an independent component filter is selected to generate the maximum transient independent signal available in the electrode data. Basically, the source of information in the data contaminated with noise has been recorded on the scalp electrodes. This contamination process is passive and linear. These sources of information can represent synchronous activity from noncortical sources (eyeball and/or muscle movement potential), as shown in Figure 2. The noise removal process using ICA is done by inspecting each channel's scalp topography and spectral power.

Eye or eyeball artifacts are almost always present in EEG recordings. They tend to be easily observed and have dominant high power in the front position on the scalp topography. The following criteria are applied in identifying a noise source containing eye movement: a smoothly decreased EEG spectrum is typical of ocular artifacts, and scalp topography shows high-power frontal projections.

An example of an EEG wave contaminated by eye movement or blinking is shown in Figure 3 in the following. The red color in the front area indicates high power. This component is eliminated and becomes a reference for other channels to get the original signal information that is not contaminated by eye movement noise.

Figure 2 also shows the T3 channel, which is thought to be contaminated with muscle noise. Furthermore, the inspection was carried out through topographic and spectral plots, as presented in Figure 4.  Figure 4(a) shows the scalp topography, with dominant energy in the area around the left ear associated with the jaw muscles. This is confirmed by a spectral plot showing the dominant activity at high frequencies (>30 Hz), as presented in Figure 4(b).

Meanwhile, line noise has a topography like muscle noise, and it always comes with high power. This noise will be easier to identify using the power spectral.  Figure 5 shows the topography and spectral power in one of the channels contaminated with line noise, where the dominant power is found at a frequency of 50 Hz.

The article "EEG-Based Spectral Dynamic in Characterization of Poststroke Patients with Cognitive Impairment for Early Detection of Vascular Dementia" was published in 2022. Journal: J Healthc Eng.

This inspection is carried out visually by observing all EEG recordings and eliminating noise-containing channels. Furthermore, signal filtering in the range of 1–30 Hz is carried out to represent the existence of the delta, theta, alpha, and beta bands. A high-pass filter with a cut-off of 1 Hz and a low-pass filter with a cut-off of 30 Hz based on IIR Butterworth were employed in this stage.

### 2.4. Spectral Dynamics Estimation Using Entropy

Generally, entropy is a measurement of signal complexity [23]. The higher the entropy value represents the more unpredictable the system. In this study, signal complexity is calculated using spectral entropy. SpecEn represents the probabilities of power spectral. SpecEn describes the spectrum irregularities of the signal in the frequency domain [24]. SpecEn estimates the change in the amplitude component of the EEG spectral power as a probability calculated using Shannon's entropy [25]. The spectral entropy is normalized according to the frequency range [*f*1, *f*2], as shown in the following equation.

(1) $$\begin{array}{c} SE\left[f1,f2\right]=-\frac{1}{\log\;\left[N\left[f1,f2\right]\right]}\overset{f2}{\underset{fi=f1}{\sum }}P_{n}\left(f_{i}\right)\log\;\left(P_{n}\left(f_{i}\right)\right)\text{,} \end{array}$$

where *s*[*N*[*f*1, *f*2]] is the total components of frequency in range [*f*1, *f*2] and *P*_*n*_(*f*_*i*_) is the probabilities of the total components of frequency [26, 27]. Higher SpecEn values indicate more complex signals, as illustrated in Figure 6.

### 2.5. Significance Test Using Statistical Analysis

Since the number of samples is small, the validation of the proposed method is carried out through statistical analysis by calculating the significance level. This test was used to observe whether there were statistically significant differences in SpecEn between groups. This study calculated the significance test using one-way variance analysis (ANOVA) and post hoc multiple comparisons based on the Tukey approach for a more detailed difference test. We set a 95% confidence level. Significance was calculated for each electrode and was considered significant if it generated a *p* value <0.05.

## 3. Results

In this section, the results of each signal processing stage are discussed in detail and followed by a discussion.  Figure 7 shows the results of denoising ICA from one of the EEG recordings after the noise source channel is eliminated. Channel-1 and channel-5 show the signal after eye noise compensation. Meanwhile, signal correction after muscle noise elimination was found in channel-3.  Figure 8(a) shows the scalp topography validation of channel-1 after eliminating the noise component.  Figure 8(b) shows the power spectral of channel-3 after the elimination of muscle noise. From the topography, it can be seen that there is no high-power spectral in the frontal area. Re-evaluation in this stage is performed on all EEG recordings to ensure the EEG signal is free of noise. In the next stage, the EEG signal is filtered to get a signal with a frequency of 1–30 Hz, followed by SpecEn measurements.

The article "EEG-Based Spectral Dynamic in Characterization of Poststroke Patients with Cognitive Impairment for Early Detection of Vascular Dementia" was published in 2022. Journal: J Healthc Eng.

The average results of SpecEn measurements on 19 channels for each group are presented in Figure 9. These results indicate that poststroke patients with cognitive impairment tend to have lower spectral complexity than the normal group. It indicates a decrease in the spectral power dynamics of the EEG signal. Moreover, it was also found that there was a relationship between the degree of signal complexity and the severity of cognitive impairment, as the results of the study reported by Al-Qazzaz [18, 19]. Patients with dementia generate lower SpecEn than patients with mild cognitive impairment SpecEn. Measurements in the 1–30 Hz range generated significant differences compared to the previous study by Al-Qazzaz et al. [19], which calculated SpecEn in the 1–60 Hz range.

Furthermore, validation is carried out with a significance test. The results of the ANOVA test are presented in Table 2. Different tests that generated *p* value <0.05 showed significant differences between groups. The results of ANOVA with a *p* value <0.05 were found for all electrodes.

Post hoc multiple comparisons with Tukey's approach were then performed to confirm the significance between groups, including normal vs. stroke-MCI, normal vs. stroke-dementia, and stroke-MCI vs. stroke-dementia. The results of the multiple comparison tests are presented in Table 3. The post hoc test results showed a significant difference between the pairs of groups found on the F7. The post hoc test results also showed that statistically, there was a significant difference in normal vs. stroke-dementia cases. Meanwhile, in normal vs. stroke-MCI and stroke-MCI vs. stroke-dementia cases, significance was found in several EEG channels. It can be thought of, and in the case of comparison, the EEG signal has a very smooth change and has similar characteristics.

## 4. Discussion

The brain represents a dynamic system that is nonlinear, nonstationary, and complex. The degree of complexity is considered to be able to represent the condition of the brain, referring to the dynamic nature of the brain [28]. This study showed that the EEG waves in the cognitively impaired group tended to have lower spectral dynamics than the normal group, as reported in the study by Nobukawa et al. [29]. In other terms, EEG signals in the pathology group had a lower degree of irregularity or less complex electrophysiological behavior than in the normal group.

The article "EEG-Based Spectral Dynamic in Characterization of Poststroke Patients with Cognitive Impairment for Early Detection of Vascular Dementia" was published in 2022. Journal: J Healthc Eng.

Changes in brain dynamics, represented as degrees of complexity in the cognitive impairment group, can be related to neuronal cell death followed by a decrease in brain functional coupling so that neural dynamics are disrupted [30]. Impaired brain functional connectivity will lead to brain failure to integrate electrophysiological networks between brain areas, which can underlie cognitive function changes.

EEG complexity studies in cases of patients with poststroke MCI and dementia show the same characteristics as AD. The results of the complexity calculation on the EEG recording of memory activity showed that the poststroke patient group with cognitive impairment tended to have a lower signal complexity than the normal group (SpecEn_Dem._ < SpecEn_MCI_ < SpecEn_Normal_). Another finding from observing SpecEn values is that there is a relationship between decreased signal complexity and dementia severity, as reported in the study by Al-Qazzaz et al. [18]. This finding confirms the results of previous studies that are worsening of dementia will be followed by a decrease in signal complexity. Post hoc test results in normal vs. stroke-dementia showed significant differences in all brain areas. This finding confirms the studies by Al-Qazzaz et al. [18] and Musa et al. [31], which interpreted the characteristic differences to be significant between normal and VaD. Their study yielded 100% and 94.4% accuracy in cases classified as normal and VaD, respectively. It is hoped that if the SpecEn feature is used in the automatic classification simulation, it is expected to produce high detection accuracy, especially in normal and stroke-dementia cases. Interestingly, and it should be noted that the proposed study found a significant difference in SpecEn values between groups on the F7-channel, which is considered to represent the frontal area. The frontal area is strongly associated with executive function [32], which is common in patients with VaD [33]. Executive function deficits appear in early or mild vascular dementia [34]. Analysis of EEG signal patterns in the frontal area can be an exciting topic in the early detection of vascular dementia.

SpecEn shows a change in the frequency distribution of the power spectrum. This is related to slowing the EEG waves in MCI and dementia patients [28, 35]. The most likely physiological interpretation to explain this is the occurrence of significant brain cholinergic deficits as the basis for symptoms of cognitive decline [36]. Cholinergic regulates spontaneous activity at low frequencies, followed by the loss of neurotransmitters and slowing nerve oscillations.

The article "EEG-Based Spectral Dynamic in Characterization of Poststroke Patients with Cognitive Impairment for Early Detection of Vascular Dementia" was published in 2022. Journal: J Healthc Eng.

The findings of this study suggest that the analysis of EEG spectral dynamics can be a method to investigate and differentiate dementia in poststroke patients. It is also hoped that it can be used to determine the severity of poststroke dementia so that it can be used for early detection. Future studies need to be extended to a larger population to meet the statistical criteria that can be considered to support a clinical diagnosis. The simulation in this study can provide knowledge that each group has discriminant characteristics. The proposed method can simplify the detection process with an automatic classification algorithm as a complement to validation in clinical diagnosis.

## 5. Conclusions

In this study, we investigated the EEG signal as a proposed biomarker for the diagnosis of poststroke dementia. This study involved forty-two participants, consisting of sixteen normal subjects, fifteen poststroke patients with mild cognitive impairment, and eleven poststroke dementia patients. Signal characterization was performed using spectral entropy (SpecEn) to measure the irregularity of the EEG spectral power, which was thought to be correlated with cognitive impairment. From the results of the SpecEn calculation, it is known that the cognitive impairment group tends to generate a lower SpecEn than the normal group, which means it has lower complexity than the normal group EEG. One-way ANOVA showed a significant difference with *p* < 0.05 between normal and cognitive impairment found in all EEG channels. Post hoc test confirmed the relationship between signal complexity and the severity of dementia where SpecEn_Dem._ < SpecEn_MCI_ < SpecEn_Normal_. From this test, there were significant differences between groups on the F7-channel. Meanwhile, in normal vs. poststroke MCI and poststroke MCI vs. poststroke dementia cases, significant differences were found in different channels.

The results of this study indicate that the measurement of the spectral complexity of the EEG signal has the potential to be a discriminatory feature between normal subjects and poststroke patients with cognitive impairment. It is also expected to be used to evaluate the severity and early detection of vascular dementia. However, spectral entropy is sensitive to noise so the processed EEG signal must be free from low- and high-frequency noise to avoid measurement errors. Another issue is that, this study is still limited in the number of samples. The next study is to increase the number of samples, explore other complexity methods to obtain higher feature gaps between groups, and continue with performance validation of the proposed method through classification simulation to determine the accuracy of the proposed method.

The article "EEG-Based Spectral Dynamic in Characterization of Poststroke Patients with Cognitive Impairment for Early Detection of Vascular Dementia" was published in 2022. Journal: J Healthc Eng.

## Figures and Tables

**Figure 1:** EEG processing stage in this study.

**Figure 2:** Example of an EEG signal contaminated with noise.

**Figure 3:** Scalp topography in a channel that is strongly suspected of containing eye movement noise.

**Figure 4:** (a) Scalp topography in the channel is suspected of containing muscle noise and (b) it is spectral.

**Figure 5:** (a) Scalp topography (b) spectral power in the channel suspected of containing line noise.

**Figure 6:** Two signals with different complexity (a) SpecEn = 0.5754 (b) SpecEn = 0.997.

**Figure 7:** ICA-based denoised EEG signal.

**Figure 8:** (a) Scalp topography after eye noise elimination (b) power spectral of channel-T3 after muscle noise elimination.

**Figure 9:** Mean SpecEn of each group.

**Table 1:** Demographic data of the control group and patient.

Index	Normal	Poststroke no dementia (MCI)	Poststroke dementia
Number of samples	16	15	11
Sex (M/F)	8/8	7/8	6/5
Age (std. dev.)	57.18 ± 4.16	59.82 ± 6.41	60 ± 5.34
Education (year)	13.45 ± 3.44	12.18 ± 4.11	14 ± 3.89
Onset stroke (month)	—	11.55 ± 7.22	17.75 ± 9.55
MoCA-INA	26.5 ± 0.67	22.33 ± 2.10	12.38 ± 4.37

**Table 2:** Significance test results for each EEG channel.

Channel	*F*-statistic	*P* value
Fp1	6.662	0.0032
F7	13.1172	≤0.001
T3	9.4634	≤0.001
T5	6.4278	0.0039
Fp2	6.6593	0.0033
F8	10.0087	≤0.001
T4	10.8629	≤0.001
T6	10.5156	≤0.001
F3	12.009	≤0.001
C3	8.8403	≤0.001
P3	5.4087	0.0084
O1	3.8516	0.0298
F4	11.3396	≤0.001
C4	11.248	≤0.001
P4	8.2756	≤0.001
O2	7.0931	0.0024
Fz	10.0438	≤0.001
Cz	6.7725	0.003
Pz	4.1805	0.0226

**Table 3:** Significant test results of multiple comparisons.

Comparison	Significant (95% confidence level)																		
	Fp1	F7	T3	T5	Fp2	F8	T4	T6	F3	C3	P3	O1	F4	C4	P4	O2	Fz	Cz	Pz
Normal vs. stroke-MCI	0.141	0.047 ^*∗*^	0.207	0.108	0.247	0.071	0.144	0.030 ^*∗*^	0.079	0.173	0.207	0.262	0.042 ^*∗*^	0.19	0.148	0.213	0.011 ^*∗*^	0.020 ^*∗*^	0.17
Normal vs. stroke-dementia	0.002 ^*∗*^	≤0.001 ^*∗*^	≤0.001 ^*∗*^	0.003 ^*∗*^	0.002 ^*∗*^	≤0,001 ^*∗*^	≤0 001 ^*∗*^	≤0.001 ^*∗*^	≤0.001 ^*∗*^	≤0.001 ^*∗*^	0.006 ^*∗*^	0.024 ^*∗*^	≤0.001 ^*∗*^	≤0.001 ^*∗*^	≤0.001 ^*∗*^	0.002 ^*∗*^	≤0.001 ^*∗*^	0.004 ^*∗*^	0.020 ^*∗*^
Stroke-MCI vs. stroke-dementia	0.174	0.020 ^*∗*^	0.026 ^*∗*^	0.251	0.097	0.062	0.019 ^*∗*^	0.11	0.020 ^*∗*^	0.044 ^*∗*^	0.232	0.395	0.054	0.011 ^*∗*^	0.071	0.09	0.315	0.154	0.513

^*∗*^*p* value <0.05.

## Data Availability

Accesses to data are restricted due to ethical approval and patient confidentiality but for research purposes, it is available from the corresponding author upon reasonable request.
